# Effects of replacing groundnut cake with rumen content supplemented with or without enzyme in the diet of weaner rabbits

**DOI:** 10.1186/s12944-015-0158-3

**Published:** 2015-12-18

**Authors:** A. A. Adeniji, S. Rumak, R. A. Oluwafemi

**Affiliations:** Department of Animal Science, Faculty of Agriculture, University of Abuja, P.M.B 117, FCT-Abuja, Nigeria

**Keywords:** Rabbits, Groundnuts cake, Rumen contents and enzyme

## Abstract

**Background:**

Rabbits are also herbivores which efficiently convert fodder to food. They are prolific and converter of plant proteins of little or no use to people as food into high-value animal protein. Rabbit meat is high in protein, low in calories and low in fat and cholesterol contents, being considered as a delicacy and a healthy food product. Feeding rabbits with concentrates is expensive and therefore in order to reduce cost of production, hence the use of rumen content in this study as alternative feedstuff without competition.

**Methods:**

A total of thirty six (36) weaner rabbits *(oryctalagus cuniculus)* of different body weight and age where use in this experiment to determine the effects of replacing rumen content with or without enzyme supplementation for groundnut cake. This feeding trial which lasted for 8 weeks was carried out in order to determine the replacement value of groundnut cake with rumen content with or without enzyme in the diet of weaner rabbit. A 3x2 factorial experiment was adopted such that there where three (3) replacement level of rumen content (0, 25 and 50 %) for groundnut cake by two supplemental level (no enzyme and enzyme supplement).

**Results:**

The results showed that increased inclusion level of rumen content has significant effects (*p* < 0.05) on daily feed intake, rate of weight gain, feed to gain ratio, nitrogen retention, faecal nitrogen, total nitrogen output and nitrogen digestibility. The weight gained by rabbits fed on 0, 25 and 50 % were all comparable (*p* > 0.05) with weight gained value of 7.62,7.44 and 7.36 g respectively. Similarly there was a significant (*p* < 0.05) effect of supplement added on the body weight gain of the experimental animals. There was significant effect (*p* < 0.05) of the diet on the obtained feed to gain ratio. However, there was no significant effect (*p* > 0.05) of the treatment on urinary nitrogen. Significant (*p* < 0.05) effects of supplementation was observed on the feed intake, weight gain, feed to gain ratio, faecal nitrogen, nitrogen retention and nitrogen digestibility but there was no significant effects (*p* > 0.05) of the supplementation on the nitrogen intake. The interaction between the varying levels of rumen content supplementation had significant effects (*p* < 0.05) on the feacal nitrogen, feed intake and feed to gain ratio but no significant (*p* < 0.05) effects on interaction of nitrogen intake.

**Conclusion:**

In conclusion, since the results from this study showed no negative effects on the performance of the experimental animals, the test ingredient can be used as alternative feedstuff at a lower inclusion level so as to reduce production cost and expand rabbit production.

## Background

Rabbits are also herbivores which efficiently convert fodder to food. They are prolific and converter of plant proteins of little or no use to people as food into high-value animal protein. In an efficient breeding, rabbits convert up to 20 % of the protein consumed in meat, more than for pigs (15–18 %) and cattle (9–12 %) [1]. Rabbit meat is high in protein, low in calories and low in fat and cholesterol contents, being considered as a delicacy and a healthy food product, easy to digest, indicated in feeding children and old people [2]. Rabbit meat is one of the best white lean meats available on the market, very tender and juicy. There is no religious taboo or social stigma regarding the consumption of this meat.

In Nigeria, rabbit production is considered a part time venture hence majority of rabbit production are mainly family own with small number of stock. Commercial productions are very rare and so the full potentials of rabbit are yet to be harnessed. Considering the economic and nutritional benefits of rabbit production which has been severally studied and confirmed, rabbit production need to be encouraged even now that Nigeria is in search of economic recovery strategies.

The major cost in any livestock production is feed thus feeding cost is a major problem facing rabbit production. Conventional protein feedstuffs such as soya bean meal, groundnut cake, and fish meal are quite expensive. The high cost of these ingredients has resulted in the poor feeding of rabbit. The need to source for alternative feedstuff (unconventional) so as to reduce high cost of livestock production cannot be overemphasized. Rumen content (RC) is obtained from the abattoir after slaughtering of animal. They are discarded as waste and cannot be consumed by human.

There has been a tremendous increase in interest and use of various types of dietary enzymes in swine diets to improve nutrient digestibility in recent years. Enzymes are biologically active proteins that break specific chemical bonds to release nutrients for further digestion and absorption. Enzymes that breakdown proteins are called proteases, lipases breakdown fats, and there are several carbohydrases that breakdown carbohydrates to allow them to be better digested and absorbed as energy sources [3]. Feed stuffs including unconventional ones used in animal feeding is composed of plant material, cereal and vegetable proteins which cannot be fully digested and utilized by animals, hence the need for enzyme supplementation which is known to assist in feed utilization and digestion.

## Method

### Experimental site

The experiment was carried out at the rabbitary unit of the department of Animal Science, Faculty of Agriculture, University of Abuja farm, Federal Capital Territory (FCT) (Table 1).

**Table 1:** Composition of experimental diet (Kg/100 kg)

	Levels of rumen content replacement for groundnut cake (%)					
	0 %		25 %		50 %	
Ingredients	T1	T2	T3	T4	T5	T6
Rumen content	0	0	4.5	4.5	9	9
GNC	18	18	13.5	13.5	9	9
Enzyme	0	+	0	+	0	+
Maize	40	40	40	40	40	40
Fishmeal	1	1	1	1	1	1
Maize offal	14	14	14	14	14	14
Rice bran	7.3	7.3	7.3	7.3	7.3	7.3
Wheat offal	14.2	14.2	14.2	14.2	14.2	14.2
Bone meal	3	3	3	3	3	3
Limestone	1.7	1.7	1.7	1.7	1.7	1.7
Salt	0.35	0.35	0.35	0.35	0.35	0.35
Premix	0.25	0.25	0.25	0.25	0.25	0.25
Lysine	0.10	0.10	0.10	0.10	0.10	0.10
Methionine	0.10	0.10	0.10	0.10	0.10	0.10
Total	100	100	100	100	100	100
Analyzed proximate values						
Crude protein (%)	17.57	17.57	16.31	16.31	15.08	15.08
Crude fiber (%)	5.51	5.51	7.13	7.13	8.73	8.73
Ether extract (%)	4.52	4.52	4.37	4.37	4.23	4.23
M.E cal/kg	2701.40	2701.40	2685.35	2685.35	2669.09	2669.09
Moisture (%)	8.61	8.61	8.57	8.57	8.54	8.54
Total Ash	12.28	12.28	12.77	12.77	11.95	11.95

BioMix Grower (BIOORGANICS) Primix used contained the followingper kg:VitA = 8,000,000 IU

VitD3 = 1,500,000,vitE = 7000 mg, vitk = 1500 mg, vitB1 = 2000 mg,vitB2 = 2500 mg,Niacin = 15,000 mg

pentatonicacid = 5500 mg,VitB6 = 2000 mg,VitB12 = 10 mg, folicacid = 500 mg, BiotinHg = 250 mg

cholinechloride = 175,000 mg,cobalt = 200 mg,copper = 3000 mg,iodine = 1000 mg, iron = 21,0000 mg

manganese = 40,000 mg, selenium = 200 mg, zinc = 31,000 mg, Antioxidant = 1250 mg

*Recommended inclusion level of enzyme: Enzyme: Maxi grain: 4 kg/tone of feed (0.4 g/100 kg)

Source: Field research at The teaching and research Farm, University of Abuja

### Experimental animals and their management

Thirty six weaner rabbits of mixed breeds averaging 0.2 kg- 0.3 kg body weight and aged 5 weeks were purchased from NAPRI (National Animal Production Research Institute Zaria). The rabbits on arrival at the experimental site were housed in a metal hutch with wire mesh at the base for easy collection of feaces and urine. The hutches were disinfected before the rabbits were introduced and they were given anti-stress with antibiotics for seven days and allowed to adapt to the environment.

The rabbits were randomly allocated to six (6) dietary treatments with two (2) rabbits per replicate and each treatment had three (3) replicates. During the experiment, fed and water were supplied ad-libitum throughout and the performance of the animals were monitored. Quantity of feed consumed was monitored daily for the 8 weeks trial period by taking note of the difference between feed served and feed left after 24 h. The rabbits were also weighed on weekly basis during this period to determine weight gain. The hutches were cleaned on daily basis throughout the experimental period. Feeders and drinkers were made available in each hutch since experimental animals were housed and fed differently.

### Experimental design

The rabbits were allocated to six (6) dietary treatments in a Completely Randomized Design (CRD) each treatment had three (3) replicates with two rabbits per replicate. Each rabbit was fed *adlibitum* diet and water for the eight (8) weeks study period. The six experiment diets had rumen content replacing GNC at 0, 25, 50 % dietary levels.

### Parameter / data collected

The performance of the rabbits was monitored, the initial live weight of the rabbits were recorded at commencement of the experiment, weekly weight and daily feed intake were recorded, while feed to gain ratio were also recorded and cost implication were calculated. During the last week of the study (the 8^th^ week), the faeces and the urine of the rabbits were collected by the total faeces collection and the urine method and the nitrogen in it was analyzed. The nitrogen digestibility was also calculated.

### Chemical analysis

Proximate analysis was conducted using the method of Association of Official Analytical Chemist (AOAC) [4]. Sample of the test diets and faeces were analyzed for the proximate constituents using the method.

### Data analysis

All data obtained were subjected to analysis of variance (ANOVA) using factorial design of Completely Randomized Design (CRD) Model and significant differences between means were separated using Duncan Multiple Range Test [5].

## Results

The results of the growth performance characteristics measured are presented in Table 2. The result showed that the feed intake of 50.85 g/rabbit/day in rabbit fed 0 % rumen content level was significantly higher (*p* < 0,05) while rabbit fed on 25 % rumen content had an intake of 50.04 % which is significantly (*p* < 0.05) higher than 49.79 g consumed by rabbit fed 50 % rumen content. Rabbits fed on enzyme supplemented diet had a higher feed intake value (50.26 g) when compared with rabbits fed on experimental diets without enzyme which had 50.19 g.

**Table 2:** Growth performance characteristics of weaner rabbits fed rumen content with or without enzyme supplementation in replacing groundnut cake

	Initial weight (g)	Final weight (g)	Daily feed intake (g)	Rate of gain (g/day)	Feed to gain
ratio					
Levels of Rumen content (%)					
0	725.00^a^	1152.00^a^	49.79^c^	7.52^a^	6.72^a^
25	675.00^b^	1091.00^b^	50.10^b^	7.44^b^	6.78^b^
50	650.00^c^	1062.00^c^	50.45^a^	7.36^c^	6.90^c^
SEM	33.0945	39.5609	0.4801	0.1163	0.0274
Significance	*	*	*	*	*
Supplements					
No Supplement	675.00^b^	1108.33^a^	50.19^b^	7.44^b^	6.80^a^
Added (NSA)					
Enzyme	691.00^a^	1096.67^b^	50.26^a^	7.50^a^	6.72^b^
(Maxigrain)					
SEM	9.1524	6.9342	0.0394	0.0394	0.0394
Significance	*	*	*	*	*
Rumen content Supplement	*	NS	*	*	*
(interaction)					

Treatment means with different superscripts along the same column are significantly different (*P* < 0.05)

NS- No significantly different (*P* > 0.05)

SEM- Standard Error of mean

Means with different superscripts (a,b,c) along the same column are significantly different (P < 0.05)

The weight gained by rabbits fed on 0, 25 and 50 % were significantly dofferent (*p* < 0.05) with weight gained value of 7.62,7.44 and 7.36 g respectively. Similarly there was a significant (*p* < 0.05) effect of supplementation on the observed body weight gain value obtained by the experimental animals. There was also significant effects (*p* < 0.05) of the diet on the obtained feed to gain ratio. The rabbits fed 0 % rumen content diets had the best feed to gain ratio of 6.72 g when compared with rabbits on other experimental diets. Rabbits fed experimental diet containing 50 % rumen content had the poorest feed to gain ratio of 6.90 g when compared with rabbits on other experimental diets.

The nitrogen intake of 3.58 g/rabbit/day (Table 3) from the experimental animals fed on the control diet was significantly higher (*p* < 0.05) than those fed on other rumen content levels. The experimental diets had no significant effect (*p* > 0.05) on nitrogen intake between the experimental animals fed enzyme and non enzyme supplemnted diets. The feacal nitrogen of rabbits fed on control diet (2.29 g/rabbit/day) was significantly higher (*p* < 0.05) than those fed on 25 and 50 % rumen content level that had 2.26 g/rabbit/day and 2.23 g/rabbit/day respectively. Similarly there was no significant (*p* > 0.05) effect of supplementation no the observed feacal values obtained on the experimental rabbits.

**Table 3:** Nitrogen digestibility of weaner rabbits fed rumen content with or without enzyme supplementation in replacing groundnut cake

	Nitrogen	Feacal	Urinary	Total nitrogen	Nitrogen	Nitrogen
	intake (g/day)	Nitrogen (g/day)	Nitrogen	Output	retained (g)	digestibility (%)
Levels of Rumen content (%)						
0	3.58^a^	2.29^a^	0.47^a^	0.49^a^	1.24^c^	63.97^c^
25	3.53^b^	2.26^b^	0.45^a^	0.45^b^	1.26^b^	64.21^b^
50	3.51^c^	2.23^c^	0.46^a^	0.41^c^	1.29^a^	64.96^a^
SEM	0.0113	0.0065	0.0033	0.0052	0.0053	0.0158
Significance	*	*	NS	*	*	*
Supplements						
NSA	3.54^a^	2.29^a^	0.46^a^	0.43^b^	1.24^b^	64.37^a^
Enzyme	3.53^a^	2.26^b^	0.47^a^	0.48^a^	1.27^a^	64.33^b^
(Maxigrain)						
SEM	0.0043	0.0097	0.0037	0.0058	0.0057	0.0873
Significance	NS	*	NS	*	*	*
Rumen content*Supplement	NS	*	NS	*	*	*

*SEM*- Standard Error of mean

Means with different superscripts along the same column are significantly different (*P* < 0.05)

NS- Not significantly different (*P* > 0.05)

SEM- Standard Error of mean

Means with different superscripts (a,b,c) along the same column are significantly different (P < 0.05)

The nitrogen digestibility of 64.96 % in weaner rabbits fed on 50 % rumen content diet was significantly higher (*p* < 0.05) than those fed on 0 and 25 % rumen content level that has 63.97 and 64.21 % respectively. Similarly there was significant (*p* < 0.05) effect of supplementation on the observed nitrogen digestibility of the experimental animals.

## Discussion

The variation in weight gain per day at different level of rumen content inclusion in the study is in conformity with several reports which indicated that rate of gain reduces with increased amount of crude fibre in the diets of monogastric animals [6]. This result contradicts the results of [7] who reported no significance difference (*P* > 0.05) when rumen content was replaced with soya beans in the diet of broiler finisher.

The significant increase (*P* < 0.05) in feed intake as the level of rumen content increased from 0 to 50 % could be because animal consumes more feed to meet its energy requirement. Also, it may be because rabbit being a pseudo-ruminant tolerates considerable level of fiber in their diet [8]. The significant increases in daily feed intake and non-significant difference in daily weight gain observed in this work agree with the results of [9] who fed bovine rumen content and reported that increasing the RC level in the diets significantly increased feed consumption but with non-significant difference in growth rate. Alawa and Umunna [10] stated that the inclusion of agro-industrial by products in livestock rations has often resulted in increased feed intake as a compensation for the reduced energy concentration of such diets. In terms of supplement, rabbits fed enzyme supplemented diets are significantly (*p* < 0.05) better than rabbits fed no supplement. This may be because enzyme increases the intake of feed.

The utilization of feed decreased from 0 to 50 % inclusion level of rumen content. This result is in agreement with the reports of [11] who reported significant effects of blood rumen content on poultry but did conform with the reports of [9] who fed rabbit with rumen content. In term of supplement, rabbit fed enzyme supplemented rumen content had better feed utilization compared with rabbit fed no supplement. The significant increase in feed to gain ratio in this study is in contrast with the work of [12] who replaced maize with rumen content in the diet of a weaner rabbit.

The result showed that the nitrogen intake increased as the level of rumen content increased. The difference in the nitrogen intake could be attributed to the difference in the crude protein contents of the diets. This result contradicts the work reported by [12] who observed insignificance difference when rumen content maggot meal mixture was fed in the diet of early weaned piglet. In terms of supplement, the result showed that there were higher values of nitrogen intake in rabbit fed with enzyme supplementation when compared to rabbits fed no supplement. This may be because of the activity of enzyme in the diet.

There was significant increase in the nitrogen digested with increase in the level of rumen content. This may be as a result of crude protein content of the diet. This is in contrast with the findings of [12] who reported no significant difference in the nitrogen digested with the increase in the inclusion level of rumen content maggot meal in the diets of early weaned pig. The result showed that there were higher values of nitrogen digested in rabbit fed with no supplementation as compared to those fed enzyme supplementation. This may be as a result protein content of the diet.

There was significant difference in the nitrogen digestibility as observed with varying levels of rumen content. This may suggest that the crude fibre contents in all the dietary treatment were different and therefore, did affect the digestibility of the rabbits. However, other reports which contradict this result indicated that nitrogen digestibility was lowered with increase in the level of rumen content [12].

## Conclusion

In conclusion, since the results from this study showed no negative effects on the performance of the experimental animals, the test ingredient can be used as alternative feedstuff at a lower inclusion level so as to reduce production cost and expand rabbit production.

## References

[1] Suttle NF (2010). Mineral nutrition of livestock.

[2] Dalle Zotte A (2000). Main factors influencing the rabbit carcass and meat quality.

[3] Xu G (2008). The role of feed enzymes in swine feeding programs.

[4] A.O.A.C (1990). Association of official analytical chemists.

[5] Steel RG, Torrie JH (1980). Principles and procedure of statistics.

[6] Numbela ER (2001). Effect of replacing palm kernel cake with rice husk in the diets of growing pigs. Animal Prod J Vol.

[7] Onu PN, Otuma MO, Odukwe CA, Aniebo AO (2011). Effects of different levels of bovine rumen content on productive performance, carcass characteristics and economics of production of finisher broilers. Int J Food Agric Vet Sci.

[8] Aduku OA, Dim NI, Aganga AA (1988). Note on a comparative evaluation of palm kernel cake, peanut and sun flower meal in the diets of weaning rabbits. J Applied Rabbit Res.

[9] Dairo FAS, Aina OO, Asafa AR (2005). Performance evaluation of growing rabbits fed varying levels of rumen content mixture. Nig J Anim Prod.

[10] Alawa JP, Umunna NN (1993). Alternative feed formulation in developing countries: Prospects for utilization of Agro-Industrial by-products. J Anim Prod Res.

[11] Adeniji AA, Balogun OO (2001). Evaluation of rumen content mixture in the diets of starter chicks. Niger J Animal Prod.

[12] Adeniji AA (2008). Replacement value of maize with enzyme supplemented decomposed bovine rumen content in the diet of weaner rabbits. J Anim Vet Adv.

